# A modified multilocus sequence typing protocol to genotype *Kingella kingae* from oropharyngeal swabs without bacterial isolation

This article has been retracted.

**DOI:** 10.1186/s12866-017-1104-5

**Published:** 2017-09-21

**Authors:** Nawal El Houmami, Janek Bzdrenga, Jean-Christophe Pons, Philippe Minodier, Guillaume André Durand, Anis Oubraham, Dimitri Ceroni, Pablo Yagupsky, Didier Raoult, Philippe Bidet, Pierre-Edouard Fournier

**Affiliations:** 1 Aix-Marseille Univ, UM63, CNRS 7278, IRD 198, Inserm 1095, Assistance Publique – Hôpitaux de Marseille, URMITE, Institut Hospitalo-Universitaire Méditerranée Infection, 19-21 Boulevard Jean Moulin, 13385 Marseille, France; 2 University of Grenoble Alpes, CEA, CNRS, IBS, F-38000, Grenoble, France; 3 Department of Pediatric Emergency Medicine, North Hospital, Aix-Marseille University, Marseille, France; 4 Département de l’enfant et de l’adolescent, HUG-Hôpital des Enfants, Geneva, Switzerland; 5 Clinical Microbiology Laboratory, Soroka University Medical Center, Beer-Sheva, Israel; 6 Laboratoire de Microbiologie, Hôpital Robert Debré, Assistance Publique – Hôpitaux de Paris, Université Paris Diderot, Sorbonne Paris Cité, Inserm, IAME, UMR 1137, Paris, France

**Keywords:** *Kingella kingae*, MLST, Pediatrics, Outbreaks, Bone and joint infections

## Abstract

**Background:**

Outbreaks of *Kingella kingae* infection are an emerging public health concern among daycare attendees carrying epidemic clones in the oropharynx. However, genotyping of such epidemic clones from affected cases is limited by the low performance of current methods to detect *K. kingae* from blood samples and lack of specimens available from infected sites. We aimed at developing a modified multilocus sequence typing (MLST) method to genotype *K. kingae* strains from oropharyngeal samples without prior culture. We designed in silico MLST primers specific for *K. kingae* by aligning whole nucleotide sequences of *abcZ*, *adk*, *aroE*, *cpn60*, *recA*, and *gdh*/*zwf* genes from closely related species belonging to the *Kingella* and *Neisseria* genera. We tested our modified MLST protocol on all *Kingella* species and *N. meningitidis*, as well as 11 oropharyngeal samples from young children with sporadic (*n* = 10) or epidemic (n = 1) *K. kingae* infection.

**Results:**

We detected *K. kingae*-specific amplicons in the 11 oropharyngeal samples, corresponding to sequence-type 6 (ST-6) in 6 children including the epidemic cases, ST-25 in 2 children, and 3 possible novel STs (ST-67, ST-68, and ST-69). No amplicon was obtained from other *Kingella* species and *N. meningitidis*.

**Conclusions:**

We herein developed a specific MLST protocol that enables genotyping of *K. kingae* by MLST directly from oropharyngeal samples. This discriminatory tool, with which we identified the first *K. kingae* outbreak caused by ST-6 in Europe, may be used in further epidemiological investigations.

**Electronic supplementary material:**

The online version of this article (10.1186/s12866-017-1104-5) contains supplementary material, which is available to authorized users.

## Background

Outbreaks of *Kingella kingae* infections are emerging as a public health issue in daycare facilities [1–3]. Defined as the occurrence of at least two epidemiologically connected cases of *K. kingae* infections within a 1 month-period, they are characterized by a high attack rate and spread of a virulent clone among children aged from 6 to 36 months sharing the same classroom, and causing a variety of osteoarticular and soft tissue infections, and occasionally endocarditis [1–3]. Epidemiological investigation of these events implies isolation and genotypic characterization of the strain causing the outbreak. At the same time, asymptomatic daycare center attendees and staff may be colonized by this virulent strain and, thus, deemed to be at risk to develop an invasive infection and/or to serve as reservoirs and sources of further dissemination of the disease [1, 2]. However, not all colonizing strains are capable of penetrating the epithelial layer and invading the bloodstream, and it is currently recognized that worldwide outbreaks are caused by a limited number of particularly invasive clones [2–4]. Epidemiological investigations revealed that only *K. kingae* clones belonging to the hypervirulent sequence types 6 (ST-6), ST-14, ST-23, ST-25, and ST-66 have caused in the past few years outbreaks in the USA, Israel and France [2–4].

Since *K. kingae* is notoriously difficult to recover in culture, real-time polymerase chain reaction (PCR) assays have been developed during the last 10 years and gained increasing acceptance for the diagnosis of *K. kingae* infections [1, 3, 5]. These culture-independent methods exhibit higher sensitivity compared to conventional cultures, shorten the time of detection from days to a few hours, enable the diagnosis in patients being administered antibiotics, as well as identification of asymptomatic *K. kingae* carriers [2, 5].When no surgical specimen is available and blood cultures are negative, alternative strategies have been developed [1, 5, 6]. Notably, the presence of an oropharyngeal *K. kingae* carriage in children under the age of four with sporadic osteoarticular infection was demonstrated to have a 90.5% positive predictive value for *K. kingae* infection [6]. On this point, it was demonstrated that *K. kingae* clones carried in the oropharynx of children with *K. kingae* infection are genotypically identical to those detected within infected sites [7].

Although the apparent increase in reported cases of *K. kingae* infections can be partly explained by improved isolation methods and better recognition of this emerging pathogen, the drawback of molecular detection tests is that, until now, they did not enable typing of the colonizing organisms and, thus, did not distinguish between individuals carrying non-invasive *K. kingae* strains and those colonized by the strain which caused the outbreak. We herein report the development of a modified multilocus sequence typing protocol (MLST) which enables to genotype *K. kingae* in oropharyngeal samples with no prior culture. This method was applied in clinics and successfully used to investigate an outbreak of invasive *K. kingae* infection that occurred in a daycare facility in 2016 in the Marseille area (France).

## Methods

### Development of a novel specific MLST typing tool for K. Kingae

We started with the analysis of MLST primers previously described in the Institut Pasteur MLST *K. kingae* database [8], and we observed a lack of in silico primer specificity between the *Kingella* and *Neisseria* genera. Therefore, we designed specific MLST primers for *K. kingae* by using the following criteria:

1. maximizing mismatches against other *Kingella* and *Neisseria* species, especially at the 3′ end;
2. maximizing consensus between distinct *K. kingae* sequence types;
3. selecting hybridization temperatures close to 58 °C (Additional file 1: Figure S1). We designed thereafter a modified MLST method for *K. kingae*, consisting in PCR amplification and sequencing of 6 housekeeping genes, namely *abcZ*, *adk*, *aroE*, *cpn60*, *recA*, and *gdh/zwf* (Table 1). We first aligned the whole nucleotide sequences of the 6 above-mentioned housekeeping genes from fourty *K. kingae* strains, as well as those from closely-related species including, *K. negevensis* Sch538^T^ [9], *K. denitrificans* ATCC 33394^T^ *, K. oralis* ATCC 51147^T^, *N. meningitidis* Z2491*, N. lactamica* 020–06*,* and *N. elongata* subs. *N. elongata* subs. *glycolytica *ATCC 29315^T^.

**Table 1:** PCR protocol for specific *Kingella kingae* multilocus sequence typing

Primer design				
Gene	Primers name	Primers	Primer length (bp)	Amplicon length (bp)
*abcZ*	abcZ_Kki_Fwd	CGCAAGAAAGCGTGTTTGAC	20	532
	abcZ_Kki_Rev	CAATTCCTGCGCCTTTTTCTC	21	
*adk*	adk_Kki_Fwd	CACACAAGCGCAATTTATTACG	22	491
	adk_Kki_Rev	AAACTTCGGTTTGTTCGTGATAT	23	
*aroE*	aroE_Kki_Fwd	CAAATCCCCACAAATTCATCAATG	24	621
	aroE_Kki_Rev	AACGCGGTGGGCTGGTTC	18	
*cpn60*	cpn60_Kki_Fwd	CATGGGCGCACAAATGGTT	19	467
	cpn60_Kki_Rev	CAAACAACAACACAAATGGGC	21	
*recA*	recA_Kki_Fwd	GACGGCAGCCACCAAGAC	21	456
	recA_Kki_Rev	TCCTGCCAGTTTACGCAAG	19	
*gdh/zwf*	gdh/zwf_Kki_Fwd	GAGCGCGGCGAGTTTTAT	18	671
	gdh/ zwf_Kki_Rev	CAGTTGTCCAAAATTGGCATG	21	
10× PCR Buffer		1×		
25 mM MgCl_2_		2.0 mM		
dNTP mix (10 mM of each)		200 μM of each dNTP		
Forward primer		0,1 μM		
Reverse primer		0,1 μM		
HotStarTaq DNA Polymerase		2.5 units/ reaction		
Distilled water		variable		
Template DNA		< 0,5 μg		
Total volume		50 μl		
PCR protocol				
Cycle step	3 step-protocol		Cycles	
	Temperature	Time		
Initial denaturation	95 °C	15 min	1	
Denaturation	95 °C	1 min	35	
Annealing	58 °C	30 s		
Elongation	72 °C	1 min 30 s		
Final elongation	72 °C	10 min	1	

Finally, we tested this novel *K. kingae* MLST protocol on 11 oropharyngeal samples that had previously been tested positive for *K. kingae* by specific real-time PCR targeting the *cpn60* gene [10], and on DNA from *K. denitrificans* CIP 103803*, K. oralis* CIP 103473*, K. potus* CIP 108935*, K. negevensis* Sch538^T^, and *N. meningitidis* CSUR P782.

## Results

*K. kingae*-specific amplicons were detected by Sanger sequencing in all tested oropharyngeal specimens corresponding to ST-6 in 6, ST-25 in 2, and possible novel STs in 3, but in none of the strains from others *Kingella* species and *N. meningitidis* (Table 2). A few single nucleotide polymorphisms (SNPs) were detected in some alleles for 7 specimens. In these cases, the highest peak of the chromatogram was selected to determinate the dominant sequence (Fig. 1). Given that only one copy of each reference housekeeping gene was found in the *K. kingae* KWG1 genome, the only strain for which the whole genome was sequenced using the highly reliable Pacific Biosciences SMRT technology [11], we postulate that *K. kingae* clones belonging to different STs may co-exist in the oropharynx of these individuals where one clone dominated.

**Table 2:** Specific multilocus sequence typing (MLST) for *Kingella kingae* performed by Sanger sequencing method on DNA directly extracted from 11 oropharyngeal specimens (=11 children) with no prior bacterial isolation allowed to detect *K. kingae* clones belonging to ST-6 in 6 children, ST-25 in 2, and possible new STs in 3, namely ST-67, ST-68, and ST-69

No.	Age (mo)	Year	Syndrome	Country/region	*abcZ*	*adk*	*aroE*	*cpn60*	*gdh/zwf*	*recA*	ST	STc
**1572468**	**17**	**2016**	**OAI**	**France**	**5**	**2**	**4**	**5**	**5**	**1**	**6**	**6**
1980738	16	2016	OAI	France	5	2	4	5^*^	5	1	6	6
1956884	18	2016	OAI	France	5	2	4	5	5	1	6	6
1882247	16	2016	OAI	France	5	2	4	5	5	1	6	6
1815589	12	2016	OAI	France	5^*^	2	4^*^	5	5^*^	1^*^	6	6
6847254	8	2016	OAI	France	5	2	4^*^	5^*^	5	1^*^	6	6
1541670	11	2016	OAI	France	7	2	6	2	2	2	25	25
0990626	28	2015	OAI	France	7^*^	2	6	2	2	2	25	25
1822057	7	2016	OAI	France	1	2	6	2^*^	1^*^	14^*^	69	…
1730798	33	2013	AC	French Guiana	5	2	3^*^	2	2	2	68	…
1746575	8	2013	AC	French Guiana	5^*^	2	6^*^	11^*^	9^*^	1^*^	67	…

^*^: detection of SNPs *OAI* osteoarticular infections, *AC* asymptomatical carriage, *mo*: months …: not defined

Data referring to the second epidemic case of the Châteauneuf-Grasse *K. kingae* outbreak 2016 are indicated in bold

**Fig. 1:** Chromatograms illustrating single nucleotide polymorphisms that were detected in nucleotide position 150 of the allele *abcZ-5* and those identified in nucleotide 336 of the allele *gdh/zwf*-5 from oropharyngeal sample No. 1815589. In these cases, the highest peak was selected to determinate the dominant clone. The nucleotide positions refer to the corresponding allele reference numbers provided in the Institut Pasteur database (http://bigsdb.pasteur.fr/perl/bigsdb/bigsdb.pl?db=pubmlst_kingella_seqdef_public&page=downloadAlleles)

This method was then applied in clinics in 2016. The study was approved by the Ethics committee of the IHU Mediterranee-Infection under reference number 2016–024. From June to July 2016, an outbreak of *K. kingae* osteoarticular infection involving two infants (aged 17 and 19 months) who shared the same classroom was identified in a daycare facility in southern France. The first patient sustained a left ankle arthritis and the second a first metatarsophalangeal joint’s arthritis. Both had presented with herpangina, fever, and peri-oral rash in the 2 previous weeks. Blood cultures were negative and no joint fluid was surgically collected in either case. Both children recovered with no sequelae after receiving intravenous cefamandole followed by oral amoxicillin. An oropharyngeal sample from the second case was collected prior to antibiotic therapy. Detection of *K. kingae* using specific real-time PCR was positive in this specimen. By using our modified MLST typing tool, we unambiguously identified *K. kingae* belonging to ST-6 composed of *abcZ*-5, *adk*-2, *aroE*-4, *cpn60*–5, *gdh*/*zwf*-5, and *recA*-1 alleles.

## Discussion

We herein developed a specific MLST method enabling to genotype *K. kingae* in oropharyngeal samples without requiring prior strain isolation. Given the fastidious nature of the species and the increasing use of molecular techniques for investigating epidemics or sporadic infections, such an improved genotyping tool is relevant. Indeed, it was previoulsy demonstrated that the presence of an oropharyngeal invasive *K. kingae* carriage in children under four with sporadic osteoarticular infections had a 90.5% positive predictive value for *K. kingae* infection [6]. Regarding this matter, it is important to note that, of the eleven *K. kingae* outbreaks in daycare centers that have been reported to date [2, 3], only 30% of children (10/33) underwent surgical procedures to obtain synovial fluid or tissue samples. This may be explained by the fact that most infected sites during *K. kingae* outbreaks were located within small joints located in hands, wrists and feet, ankles, as well as bony sites rich in growth cartilage such as epiphysis of long bones and spine [2]. Since these are regions where joint fluids are uncommonly sampled and epiphyseal bone, vertebrae, or intervertebral disks specimens are rarely obtained, many cases remain unconfirmed [1–3] but are still treated since *K. kingae* clones carried in the oropharynx of children with *K. kingae* infection are genotypically identical to those detected within infected sites [7]. In two *K. kingae* outbreaks involving four children in Israel, no suspected cases could be formally confirmed [1, 2, 12]. In this peculiar context, the genotype of epidemic clones was obtained from *K. kingae* oropharyngeal isolates cultivated from either presumed cases or from healthy classmates sharing the same classroom [1, 12].

Blood cultures and even PCR on blood specimens are really disappointing; although skeletal system infections result from the blood-borne dissemination of the bacterium, the prerequisite bacteremic episode is short and most of the time, when a localized infection has been established, the pathogen has usually been cleared from the blood.

Moreover, given that 60% of epidemic cases are not microbiologically confirmed during *K. kingae* outbreaks, and that *K. kingae* may be difficult to isolate from polymicrobial samples even on appropriate culture media [2], this specific *K. kingae* MLST tool may be helpful when oropharyngeal swabs are the only biological samples available for genotyping, as was the case in this report. Clones belonging to ST-6 are among the most invasive and disseminated worldwide and the main cause of *K. kingae* outbreaks in Israel [2, 4]. To the best of our knowledge, we here report the first *K. kingae* outbreak caused by ST-6 in Europe. Therefore, this genotype appears to be responsible for 50% of outbreaks worldwide.

## Conclusions

This modified, specific *K. kingae* MLST tool demonstrated a high discriminatory power and may be used in further epidemiological investigations for sporadic and epidemic *K. kingae* infections.

## Additional file

Additional file 1: Figure S1. MAFFT alignment of MLST genomic regions of the *abcZ*, *adk*, *aroE*, *cpn60*, *gdh/zwf*, *recA* genes from the 40 *Kingella kingae* strains that were used in this study, and those from 6 closely related *Kingella* and *Neisseria* species. Only each distinct variant of *K. kingae* sequence types is represented. MAFFT alignment and figures were performed by using Geneious 10.2.3 (Biomatters). (PPTX 24674 kb)

## Abbreviations

CIP: Collection de l’institut pasteur
CSUR: Collection de souches de l’unité des rickettsies
DNA: Deoxyribonucleic acid
IHU: Institut hospitalo-universitaire
MLST: Multilocus sequence typing
OAI: Osteoarticular infection
PCR: Polymerase chain reaction
SMRT: Single molecule real time
SNP: Single nucleotide polymorphism
ST: Sequence type
STc: Sequence type complex
